# High diversity of *Morchella* and a novel lineage of the Esculenta clade from the north Qinling Mountains revealed by GCPSR-based study

**DOI:** 10.1038/s41598-019-56321-1

**Published:** 2019-12-27

**Authors:** Phonepaserd Phanpadith, Zhongdong Yu, Tao Li

**Affiliations:** 1 College of Forestry, Northwest A&F University, Yangling, Shaanxi 712100 China; 2 Sichuan Province Forest and Grass Seedling Station, Chengdu, 610082 China

**Keywords:** Phylogenetics, Fungal genetics

## Abstract

China is a mainland country rich in natural morel recourses, having records of half of the worldwide 61 morel phylospecies. In this study, 31 collections of ascocarps from the north Qinling Mountains, 4 collections of commercial cultivars from the south Qinling Mountains, and 3 *Morchella* mycelium clones from commercial cultivars were investigated using the genealogical concordance phylogenetic species recognition (GCPSR) method. Maximum-likelihood was employed for the construction of phylogenetic trees. A total of five phylogenetic species were found among the 38 collections, namely *Morchella* sp. Mes-8, Mes-9, Mes-13, and Mes-25, and *Morchella chensiensis* (IF556780), in addition to the false morel (*Verpa bohemica*). The identification of cultivated *Morchella* sp. Mel-2, Mel-6, Mel-10, and Mel-12 coincided with that of the commercial farms. A total of 80% (4/5) of yellow morels were new records for the Qinling region, except Mes-19; moreover, a novel monophyletic lineage, *Morchella chensiensis*, was found to be distinct from the previously reported phylospecies by single gene and combined genes analysis, thus being herein proposed as a new phylospecies. All collections from this study showed continental endemism, and all Qinling Mountains collections were grouped together in rDNA phylogenetic trees. The study provided insights on biodiversities in this key region of China.

## Introduction

True morel (*Morchella* spp.), one of estimated 1.5 million species of fungi^1^, is a popular edible mushroom that is highly valuable because of its nutritional, medicinal, and economic values. Mycophiles and gourmets around the world collect *Morchella* species, and unfortunately, these anthropic activities have caused the vegetative destruction and disappearance of some *Morchella* species before they are formally described. Although mycologists and farms have recently strived to show that morels can be commercially harvested in China, Europe, North America, and other morel-rich regions^2,3^, many species are still in danger of extinction. To develop scientifically informed conservation practices and enhance the sustainability of morel harvesting, countermeasures must be implemented by governments as soon as possible. A first effort towards such measures should involve understanding morel genetic diversity, evolutionary relationships, and geographic distribution, whereas a second effort should be finding alternative manners of meeting consumer demands, for instance, through commercial cultivation. Fortunately, some species of morels namely, *M. rufobrunnea*^4,5^, *M. importun*^6^, *M. sextelata*, and *M. eximia*^7^ have been successfully cultivated, and therefore, farmers have been able to provide fresh morels to supermarkets and dried morels via the internet at an average price of 160 $/kg^3^.

Species delimitation in *Morchella* spp., however, remains complex because of their high morphological stasis and plasticity of apothecium colour and shape. Some studies have classified *Morchella* spp. using morphological species recognition (MSR) into as many as 50 species, whereas other studies have classified the genus into 3–5^8^, 30^9^, and 50 species^10^. Nevertheless, binomials have been adequately proposed for only four species and only during the last 10 years^11^. There are currently 315 nomenclatural species of fungi, including subspecies and varieties, recorded in the fungi index database (http://www.indexfungorum.org/Names/Names.asp). A total of 30 phylospecies and fewer than five morphospecies have been recorded from China^3^, while most MSR were named by Europeans and applied in North American and Asian collections.

Nevertheless, molecular phylogenetic studies have indicated that many epithets may be synonymous species, homonymous species, or incorrectly named species, given that the majority of morel species appear to exhibit high continental endemism and provincialism in the Northern hemisphere, which is consistent with their proposed evolutionary origin in Laurasia^12^. Initially, the *Internal Transcribed Spacer* (*ITS*) *rDNA* region was used as the sole locus in most studies for assessing *Morchella* genetic diversity^13^. Although *ITS* sequences were useful for identifying 77.4% of the known phylospecies, at least 66% of the named *Morchella* sequences in GenBank were misidentified^13^. Thus, the use of multilocus DNA sequence datasets and phylogenetic species recognition based on genealogical concordance and nondiscordance was initiated and accepted by academia^12,14–16^. Currently, 61 phylospecies, including 30, 22, and 19 from China, Europe, and North America, respectively, have been resolved by employing maximum parsimony and maximum-likelihood frameworks based on genealogical concordance phylogenetic species recognition (GCPSR)^17^. Moreover, a *Morchella* Multilocus Sequence Typing (MLST) internet database (http://www.cbs.knaw.nl/morchella/) was constructed for querying *Morchella* identification based on multilocus *ITS* + *LSU* + *EF*_1*-a*_ + *RPB*_*1*_ + *RPB*_2_ datasets^13^. In this database, instead of a morphospecies name, the phylospecies names within Distance Esculenta and Distance Eleta are informally named using codes starting with Mes (for the Esculenta clade) or Mel (for the Elata clade) followed by a unique Arabic number. Since 2012, this terminology has been widely applied for *Morchella* spp. nomenclature. Mes-1–27 and Mel-1–34 are the 61 currently identified species of the genus, and the third clade of *Rufobrunnea* currently comprises three MSR species but without phylospecies^13^.

In a narrow sense, the Qinling Mountains (32°–34°N) are the headstreams of the Yangtse River and the Yellow River, comprised the boundary between North China and South China, including the Guanzhong flatland and the valley of Hanjiang River in Shaanxi Province. The Qinling Mountains are connected with the Sino-Himalayan forest subkingdom and Sino-Japanese forest subkingdom, where 17 yellow morel and 13 black morel of the total 30 *Morchella* species from China have been reported, respectively^17^. However, the study of *Morchella* from the Qinling Mountains has been limited, as only Mes-19 has been reported for the south Qinling Mountains and other three phylospecies, Mes-13, Mel-13, and Mes-21, have been reported for the Tongchuan prefecture, a northern part of the Loess Plateau^17^. In this study, 31 different *Morchella* ascocarps from the north Qinling Mountains (Shaanxi), three commercial cultivars, and four mycelium clones of commercial *Morchella* from southern areas, including a neighbour province, Sichuan, were collected and identified using GCPSR. Five partial markers were used in the analyses, namely *ITS* (*ITS*_1_*/ITS*_4_)^18–20^, partial *LSU 28S rDNA* gene (*LROR/LR*_5_)^21,22^, *RNA polymerase II largest subunit* 1 (*RPB*_1*-af*_*/RPB*_1*-cr*_)^23^, *RNA polymerase II second largest subunit* 2 (*RPB*_*2–6f*_*/RPB*_*2–7*.1*r*_)^24,25^, and *translation elongation factor 1-α* (*EF*_*1–5*2*6f*_*/EF*_1*–3ar*_). Single gene and multigene phylogenetic trees were constructed to evaluate the *Morchella* species diversity, and morphological observations of these species were performed. The study aimed to help discover the diversity of *Morchella*, and help biodiversity conservation and sustainable exploration of this famous fungus in the key ecological central of China, the Qinling Mountain.

## Results

### Multilocus amplicons

The PCR products of the 38 collections were successfully amplified, generating 1.1-kb and 0.9-kb sequence regions of *ITS rDNA* and 2*8 S LSU rDNA*, respectively. For the protein coding region amplified with the *EF*_*1–526f*_*/EF*_*1–3ar*_ primer pair, 31 of the 38 (82%) collections were successfully amplified, generating a 0.7-kb region; the amplifications of seven collections of yellow morels (QL-Y04-5, QL-Y14, QL-Y16, QL-Y20, QL-Y21, QL-Y23, and QL-Y-C) failed. For the *RPB*_*1-af*_*/RPB*_*1-cr*_ primer pair, 35 of the 38 (92%) collections were successfully amplified generating a 0.8 kb region; the amplification of three collections (QL-Y02, QL-Y14, and QL-Y23) failed. For the *RPB*_*2-6f*_*/RPB*_*27–1r*_ primers, 29 of the 38 (76%) collections were successfully amplified generating a 0.7-kb region; the amplification of nine collections (QL-Y08, QL-Y12, QL-Y14, QL-Y16, QL-Y17, QL-Y19, QL-Y23, QL-Y-D, and QL-Y29) failed. The partial sequence regions of three mycelium clones (QL-Y29, QL-Y30, and QL-Y31) were 0.75 kb, 0.7 kb, 0.7 kb, 0.65 kb, and 0.6 kb for *ITS, LSU, EF*_*1-a*_, *RBP*_*1*_, and *RPB*_*2*_, respectively.

### Phylogenetic analysis based on *ITS rDNA*

Based on the phylogenetic analysis using the *ITS* marker (152 sequences and 1805 characters), with *Verpa bohemica* to root the tree, the 38 collections from the present study were initially classified into two main clades: yellow morel and black morel. As the *ITS* marker is an intron that cannot robustly differentiate cryptic species of *Morchella*^13^, ten collections formed an ambiguous sister clade including yellow morel (QL-Y02, QL-Y04-3, QL-Y04-4, QL-Y09-1, QL-Y21, QL-Y24) and black morel (QL-Y25, QL-Y29, QL-Y30, and QL-Y31) collections (100% bootstrap support (BS); Fig. 1). Nine taxa, which included 24 of the 38 collections of yellow morel (*Esculenta* clade), were identified. Among these, five collections (QL-Y15,QL-Y23,QL-Y17, QL-Y19, and QL-Y-B) were nested within a monophyletic lineage, Mes-9 (BS of 100%); another five collections (QL-Y14, QL-Y-C, QL-Y04-5, QL-Y16, and QL-Y20) within a monophyletic group, Mes-13 (99% BS); QL-Y18 was nested together with Mes-25 (100% BS); QL-Y-D was nested together with *Verpa* sp. (false morel) (100% BS); and 13 collections were grouped as an independent subclade, annotated as *Morchella chensiensis*, putatively. A total of 3 of the 38 collections were nested in black morel (Elata clade): QL-Y26 was clustered with Mel-12 (90% BS); QL-Y27 was clustered with Mel-6 (96% BS), and QL-Y28 was clustered with *M. importuna* (Mel-10; 97% BS), all were coincided with their commercial names. The phylogenetic tree based on *LSU rDNA* and *ITS* + *LSU rDNA* was not robust as ITS tree to differentiate the *Esculenta* clade from the *Elata* clade, but they both show collections from the Qinling Mountains endemic and revaluated independently (Suppl. Figs. 2 & 3).

**Figure 1:** Phylogenetic tree based on ITS-rDNA. Note: The tree covered 152 sequences (56 phylospecies of true morels) were constructed by the maximum-likelihood (ML) method. Bootstrap values ≥50% were shown on branches. Collections of *Morchella* spp. spcies, inclusive of a *Verpa bohemica* from Qinling Mt. were marked with red dots. Phylospecies were assigned according to^12,13,16,17^ *Verpa* sp. was used as the outgroup.

### Phylogenetic analysis based on the combined *EF*_*1-a*_ + *RPB*_*1*_ + *RPB*_*2*_ dataset

The maximum-likelihood phylogenetic tree of the three-gene dataset (138 sequences and 3,695 characters) using *Verpa* sp. as an outgroup is shown in Fig. 2, and nine lineages in the sister clades (*Elata* and *Esculenta*) were found. Within the *Esculenta* clade, five subclades were identified: collections of QL-Y21, QL-Y19, QL-Y17, QL-Y15, and QL-Y-B were nested within Mes-9 subclades and were therefore annotated as Mes-9 (91% BS); collections of QL-Y20, QL-Y16, QL-Y-C, and QL-Y-04-5 (except QL-Y14 in ITS-tree) were annotated as Mes-13 (91% BS); QL-Y18 was annotated as Mes-25 (94% BS); QL-Y24 was resolved as Mes-8, however in the *ITS rDNA* phylogenetic tree, collection QL-Y24 was nested within the black morels. The other 17 collections, including 13 of the putative Qinling Mountains lineage and a sublineage from the *ITS* tree that includes QL-Y02, QL-Y04-3, QL-Y04-4, and QL-Y09-1, formed a resolved monophyletic lineage as *Morchella chensiensis* (92% BS); this clade was divergent from all of the other 27 phylospecies in *Esculent* clade^17^. We were unable to sequence these three genes for collections QL-Y14 and QL-Y23, which were therefore defined as Mes-13 and Mes-9 based on the results of the *ITS* tree, respectively.

**Figure 2:** Phylogenetic tree based on EF_1-a_ + RPB_1_ + RPB_2_. Note: The tree covered 138 sequences (62 phylospecies of true morels, *Verpa* sp) were constructed by maximum-likelihood (ML) method. Bootstrap values ≥50% were shown on branches. Collections of *Morchella* spp. species, inclusive of a *Verpa bohemica* from Qinling Mt. were marked with red dots. Phylogenetic species were assigned according to^12,13,16,17^. *Verpa* sp. was used as outgroup.

The subclade *M. chensiensis* in Fig. 2 was then further analysis by using *Verpa* as the outgroup and by maximum-likelihood method based on *EF*_*1-a*_ + *RPB*_*1*_ + *RPB*_*2*_ dataset (47 sequences and 3,592 characters), all collections of *M. chensiensis* were nested together and displayed as a monophyletic species when compared to the other *Esculenta* species in Fig. 3.

**Figure 3:** Phylogenetic tree of subclade *M. chensiensis* based on EF_1-a_ + RPB_1_ + RPB_2_. Note: The tree covered 47 sequences (10 phylospecies of true morels, and a *Verpa* sp) were constructed by maximum-likelihood (ML) method. Collections of *Morchella* spp. species, inclusive of a *Verpa bohemica* from Qinling mountain were marked with red dots. Phylogenetic species were assigned according to references^12,13,16,17^. *Verpa* sp. was used as the outgroup.

Within the Elata clade in Fig. 2, collection QL-Y28 was resolved as Mel-10 (99% BS), QL-Y26 as Mel-12 (98% BS), as same as that in ITS-tree; however, collections QL-Y25 and QL-Y27 were annotated as Mel-6 (95% BS), collections QL-Y29, QL-Y30, and QL-Y31 formed a monophyletic lineage as in the *ITS* tree but resolved as Mel-2 (100% BS). QL-Y-D was identified as *Verpa boemica* (100% BS) in the root group. All phylospecies of *Morchella* spp. herein assigned using GCPSR are shown in Table 1.

**Table 1:** Phylospecies of *Morchella* spp. assigned by GCPSR in this study.

Collection	Phylospecies	Distributions
QL-Y-D	*Verpa bohemica*	China, USA
QL-Y26	*Morchella* sp. Mel-12	USA, Turkey
Ql-Y25, QL-Y27	*Morchella* sp. Mel-6	China, USA, Turkey
QL-Y29, QL-Y30, QL-31	*Morchella* sp. Mel-2	USA, Turkey
QL-Y28	*Morchella* sp. Mel-10	China, USA, Turkey
QL-Y01, QL-Y03, QL-Y04-1, QL-Y04-2, QL-Y05, QL-Y06, QL-Y07, QL-Y08, QL-Y09-2, QL-Y09-3, QL-Y10, QL-Y12, QL-Y13	*Morchella chensiensis* P. Phanpadith & Z. Yu	Shaanxi of China
QL-Y24	*Morhella sp*. Mes-8	USA, Turkey, China
QL-Y02, QL-Y04-3, QL-Y04-4, QL-Y09-1, QL-Y15, QL-Y17, QL-Y19, QL-Y21, QL-Y23, QL-Y-B	*Morchella* sp. Mes-9	China, USA, Turkey
QL-Y04-5, QL-Y14, QL-Y16, QL-Y20, QL-Y-C	*Morchella* sp. Mes-13	China, USA, Turkey
QL-Y18	*Morchella* sp. Mes-25	China

### Morphological descriptions of the Qinling Mountains lineage (Voucher HMAS2556 256)

*Typification*: CHINA. SHAANXI PROVINCE: Guanghuojie county, alt. 1,500 m, on soil under diverse forest of *Juglans regia*, *Populus* sp., and *Quercus aliena*, 15 May 2017. A new name of *Morchella chensiensis* was registered in the Index Fungorum (IF556780). Genbank accession numbers are listed in Table 2.

**Table 2:** Collections of Morchella spp. in this study (Note: “-” means no PCR products).

Collections	Locus	GPS coordinates	Habitats/dominant plants	Accession number in NCBI				
				ITS	28 S rDNA	RPB1	RPB2	EF1-a
QL-Y01	Guanghuojie/Shaanxi	33°75′N-108°76′E	*Juglans regia*	MG911212	MG911243	MH577905	MH577845	MH577874
QL-Y02	Guanghuojie/Shaanxi	33°75′N-108°76′E	*Quercus aliena B*	MG911213	MG911244	—	MH577846	MH577875
QL-Y03	Guanghuojie/Shaanxi	33°75′N-108°76′E	*Juglans Regia orchard*	MG911214	MG911245	MH577906	MH577847	MH577876
QL-Y04-1	Heihe Forest Park/Shaanxi	34°67′N-109°79′E	*Castanea mollissima*	MG911215	MG911246	HM663434	MH577848	MH577877
QL-Y04-2	Heihe Forest Park/Shaanxi	34°67′N-109°79′E	*Castanea mollissima*	MG911216	MG911247	MH577907	MH577849	MH577878
QL-Y04-3	Heihe Forest Park/Shaanxi	34°67′N-109°79′E	*Populus tomentosa*	MG911217	MG911248	MH577908	MH577850	MH577879
QL-Y04-4	Heihe Forest Park/Shaanxi	34°67′N-109°79′E	*Populus simonii*	MG911218	MG911249	MH577909	MH577851	MH577880
QL-Y04-5	Heihe Forest Park/Shaanxi	34°67′N-109°79′E	*Larix sp*.	MG911219	MG911250	MH577910	MH577852	—
QL-Y05	Heihe Forest Park/Shaanxi	34°67′N-109°79′E	*Juglans regia*	MG911220	MG911251	MH577911	MH577853	MH577881
QL-Y06	Heihe Forest Park/Shaanxi	34°67′N-109°79′E	*Juglans regia*	MG911221	MG911252	MH577912	MH577854	MH577882
QL-Y07	Heihe Forest Park/Shaanxi	34°67′N-109°79′E	*Larix sp*.	MG911222	MG911253	MH577913	MH577855	MH577883
QL-Y08	Heihe Forest Park/Shaanxi	34°67′N-109°79′E	*Larix sp*.	MG911223	MG911254	MH577914	—	MH577884
QL-Y09-1	Heihe Forest Park/Shaanxi	34°67′N-109°79′E	*Quercus aliena*	MG911224	MG911255	MH577915	MH577856	MH577885
QL-Y09-2	Heihe Forest Park/Shaanxi	34°67′N-109°79′E	*Quercus aliena*	MG911225	MG911256	MH577916	MH577857	MH577886
QL-Y09-3	Heihe Forest Park/Shaanxi	34°67′N-109°79′E	*Quercus aliena*	MG911226	MG911257	MH577917	MH577858	MH577887
QL-Y10	Guanghuojie/Shaanxi	33°75′N-108°76′E	*Populus sp*	MG911227	MG911258	MH577918	MH577859	MH577888
QL-Y12	Guanghuojie/Shaanxi	33°75′N-108°76′E	*Populus sp*	MG911228	MG911259	MH577919	—	MH577889
QL-Y13	Guanghuojie/Shaanxi	33°75′N-108°76′E	*Larix principis-rupprechtii*	MG911229	MG911260	MH577920	MH577860	MH577890
QL-Y14	Heihe Forest Park/Shaanxi	34°67′N-109°79′E	*Larix principis-rupprechtii*	MG911230	MG911261	—	—	—
QL-Y15	Guanghuojie/Shaanxi	33°75′N-108°76′E	*Juglans regia*	MG911231	MG911262	MH577921	MH577861	MH577891
QL-Y16	Guanghuojie/Shaanxi	33°75′N-108°76′E	*Juglans regia*	MG911232	MG911263	MH577922	—	—
QL-Y17	Guanghuojie/Shaanxi	33°75′N-108°76′E	*Quercus sp*.	MG911233	MG911264	MH577923	—	MH577892
QL-Y18	Guanghuojie/Shaanxi	33°75′N-108°76′E	*Pinus tabulaeformis*	MG911234	MG911265	MH577924	MH577862	MH577893
QL-Y19	Guanghuojie/Shaanxi	33°75′N-108°76′E	*Pinus tabulaeformis*	MG911235	MG911266	MH577925	—	MH577894
QL-Y20	Heihe Forest Park/Shaanxi	34°67′N-109°79′E	*Juglans regia*	MG911236	MG911267	MH577926	MH577863	—
QL-Y21	Heihe Forest Park/Shaanxi	34°67′N-109°79′E	*Juglans regia*	MG911237	MG911268	MH577927	MH577864	—
QL-Y23	Heihe Forest Park/Shaanxi	34°67′N-109°79′E	*Quercus sp*.	MG911238	—	—	—	—
QL-Y24	Heihe Forest Park/Shaanxi	34°67′N-109°79′E	*Quercus aliena*	MG911239	MG911269	MH577928	MH577865	MH577895
QL-Y25	Lijiang/Yunnan	27°13′N-102°48′E	Commercial cultivation	MG911240	MG911270	MH663435	MH577866	MH577896
QL-Y26	Linyou/Shaanxi	34°67′N-109°79′E	Commercial cultivation	DM423878	MH468773	MH577929	MH577867	MH577897
QL-Y27	Ankang/Shaanxi	32°89′N-108°51′E	Commercial cultivation	DM423879	MH468774	MH577930	MH577868	MH577898
QL-Y28	Dayi/Sichuan	30°52′N-103°52′E	Commercial cultivation	DM423880	MH468775	MH577931	MH577869	MH577899
QL-Y29	Dayi/Sichuan	30°52′N-103°52′E	Commercial cultivation	DM423881	MH468776	MH663436	—	MH577900
QL-Y30	Dayi/Sichuan	30°52′N-103°52′E	Commercial cultivation	DM423882	MH468777	MH663437	MH577870	MH577901
QL-Y31	Dayi/Sichuan	30°52′N-103°52′E	Commercial cultivation	DM423883	MH468778	MH663438	MH577871	MH577902
QL-Y- B	Fengxian/Shaanxi	33°91′N-106°51′E	*Populus cathayana*	MG911241	MG911271	MH663439	MH577872	MH577903
QL-Y-C	Shanyang/Shaanxi	33°53′N-109°88′E	*Liriodendron chinensis*	MG911242	MG911272	MH577932	MH577873	—
QL-Y-D	Honghegu/Shaanxi	34°16′N-107°76′E	*Populus cathayana*	DM423884	MH468772	MH663440	—	MH577904

The fruit body is generally similar to that of *M. esculenta* in colour of the pits, ridges, edges, and dimensions^11^. Fruit body height is 4.09–9.10 (6.88) cm. Ascocarps are brown-whitish cream to pale-yellowish brown with irregularly arranged pits. The ridge edges are usually lighter in colour than the pits, sometimes directly cone-shaped with a rounded top or more elongated. Ascocarps are spongy and attached to the stem, 1.99–5.23 (3.78) cm long × 1.23–4.97 (2.34) cm wide. The stipe is whitish to yellowish or cream coloured, hollow inside, and straight with a club-shaped base; general dimensions: 2.24–8.21 (8.36) cm long × 2.22–5.54 (2.31) cm thick (Fig. 4A).

**Figure 4:** Morphology of *Morchella chensiensis*. (**A**) Ascocarp, (**B**) Young asci full of plasma, (**C**) Spores with gelatinous coat, (**D**) Ascospores and an open cap at the apical ascus, (**E**) Paraphyses with 2 septals and swollen at the top, (**F**) Eight parrelled ascospores in each matured ascus, (**G**) asci and paraphyses, the later is shorter.

Ascospores with gelatinous coat, parrelled in ascus (Figs. 4C,B,D), with thin-smooth walls and egg-shaped, average dimension of 16.32–19.39 (17.39) µm long × 8.66–16.21 (12.18) µm wide. Each ascus with an open cap at the apex (Fig. 3f) containing eight ascospores of long cylindrical shape, with dimensions of 130.08–193.53 (156.66) µm long × 10.72–17.71 (14.29) µm wide. Paraphyses are cylindrical, 2-septate at the base (Fig. 4E), and thin in diameter, 80.34–123.11 µm long × 4.34–10.13 µm wide; some apical paraphyses are enlarged (Fig. 4G). The sample of the Qinling lineage was deposited in the Herbarium of Institute of Microbiology, Chinese Academy of Science, under the voucher number HMAS2556256.

## Discussion

The evaluation of *Morchella* species diversity is often complicated by the plasticity of macro- and micromorphological characteristics. Multigenes are therefore important for aiding in species recognition, and they are often used instead of the morphology to identify these cryptic species^10,11,17,26^. However, phylospecies are still commonly confused with those identified using MSR. For instance, Mel-10 from different regions, defined using phylogenetic tools^12,16,17^, were assigned the MSR names *M. elata*^10^ and *M. importuna*^11,26^, respectively. Within the *Esculenta* clade, the phylogenetic species corresponding to *Morchella* sp. Mes-4^13,16,17^ were assigned to the same species, whereas its MSR names included *M. rigida*^10,26^, *M. esculentoides*^11^, and *M. Americana*^14^. Therefore, a uniform recognition of this cryptic species using GCSPR methods is highly necessary.

Morel species diversity across China was recently reported, and many nonaccepted species were resolved using GCPSR methods^3,13,17^. Only four species and one subspecies, from Europe and America, had been previously identified using MSR and given Latin names. However, approximately 30 phylospecies, including 17 yellow morels and 13 black morels, have been reported in China based on results of studies using GCPSR. Among these including those overlap taxa, 20 taxa were found in the Sino-Japanese Forest subkingdom, 17 taxa in the Sino-Himalayan Forest subkingdom, 4 species in the Tibet Plateau (Qinghai-Xizang), 4 species in the Eurasia Forest Protected Area, and a few species were discovered in other regions^3^. In Shaanxi Province where morels were collected in this study, three species (Mes-13, Mes-19, and Mes-21) of yellow morel and one species (Mel-13) of black morel were reported^17^. Only Mes-19 was sampled in the south Qinling Mountains, whereas the other three species were collected in the north Loess Plateau, Tongchuan city, a vastly different region.

We recorded nine new phylogenetic species exclusively a false morel (*Verpa bohemica*) from around the Qinling Mountains, five yellow morels, and four black morels; namely, Mes-8, Mes-9, Mes-13, Mes-25, and *Morchella chensiensis* in Distant Esculenta, and Mel-2, Mel-6, Mel-10, Mel-12 in Distant Elata. Mel-13, Mes-13, Mes-21, and Mes-19 were not found in the north Qinling Mountains, although they were represented in Shaanxi from different collection sites^13,17^. The species diversity of true morels from 21 provinces in China was studied and reviewed^17^, and Mes-9 was reported in Shangdong, Mes-13 in Yunnan and Shaanxi, and Mes-25 and Mel-6 in Yunnan. In particular, *Morchella chensiensis* was not grouped within any of the 30 species reported in China, and it was found as a monophyletic group within the Esculenta clade. However, based on the descriptions of the morphological characteristics, we found almost no difference among our yellow morel collections. Mes-8 and Mes-9 presented very small differences in their morphologies^30^, and they were regarded as cospecies when the GCPSR method was applied, species boundaries between them is still ambiguous (Fig. 2). The only morphological difference between Mes-8 and Mes-9 is the size of fruit bodies, but not pileus, stipe, asci, and ascospores, and their colours^30,31^, although their phylogenetic relationship was also determined differently^11,13,16,32^. The morphology of *Morchella chensiensis* is highly similar to that of Mes-9 regarding as the size of the fruit body, pileus, stipe, asci, and ascospore, which are mostly the same or the former is slightly smaller than the latter, however, the multigene phylogenetic analysis revealed them as different monophyletic lineages. Both Mes-13 and Mes-25 have been reported in China^12,16,17^ with paraphyses of three to five septa, more than those of Mes-9 and *Morchella chensiensis*; the latter usually has paraphyses with one or two septa at the basal level.

Within the Elata clade, the morphology of *M. sextelata* had been previously described and corresponded to the phylogenetic species Mel-6^12,26^, which was best represented by collections QL-Y25 and QL-Y27 in the single gene and multigene trees. The phylospecies Mel-10 was found again and represented by collection QL-Y28 in this study, Fig. 2. The Mel-2 was previously reported in the USA^12^ and Turkey^15^, and was first represented by collections QL-Y29, QL-Y30, QL-Y31 in China. The Mel-12 had not been previously reported from China, only from the USA^11,12^ and Turkey^27^, and was first represented by collection QL-Y26. *Verpa bohemica* (false morel) was also firstly described in China^28,29^. The monophyletic group of *Verpa bohemica* has asci that consist of two huge ascospores, unlike the true morel species (Suppl. Fig. 1). The morphology of *Verpa bohemica* (false morel) was described from specimens collected in USA^29^ and Europe. We collected it from Honghegu Forest Park in north Qinling, and GCPSR grouped it with *Verpa bohemica* (100% BS). The *Verpa* clade showed a close relationship with the true morel clade, of which it seems to be a basal clade and displayed a closer evolutionarily relationship to black morels than to yellow morels.

Interestingly, all collections from the north Qinling Mountains were endemic and formed a big clade separated from the other yellow morels from Europe and North America in LSU rDNA tree and ITS + LSUrDNA tree (Suppl. Figs. 1 & 2). The Qinling region is in the Sino-Japanese forest subkingdom region, and it was believed to be a refuge during Quaternary Glacial Relics^7^. The diverse and complex ecogeography of this region had a key role in hosting many species, including plants, animals and fungi, and it also led to the reproductive isolation of species, which then resulted in high species diversity^7^. Among the 30 phylospecies of *Morchella* spp. in China, 20 are distributed in the Sino-Japanese forest subkingdom region^3^. A total of 13 of the 17 yellow morel species and 7 of the 13 black morel species were found in this subkingdom region; however, only at the Qinling Mountains area, four new recorded species of yellow morels were discovered, and a new lineage, *Morchella chensiensis*, was resolved. The Qinling Mountains hosts a high diversity of *Morchella* spp. conclusively.

## Materials and Methods

### Collection of *Morchella*

Thirty-one fresh morels were collected under a broad-leaved forest below 1600 m altitude in the north Qinling Mountains in May 2016 and 2017. Details of each collection, including information on habitation, coordinates, and amplified loci, are listed in Table 2. Four collections and three mycelium clones of cultivated black *Morchella* from the south Qinling Mountains were also included in this study.

### Morphological description

A small portion of pileus from each sample was removed and placed on a slip glass for 4–5 min, immersed in 100 µL of water, and then sliced to10–15 nm thickness particle size by hand. The sliced samples were transferred to new slip glasses and covered with a thin cover slip, which was pressed to spread the sample. The morphological assessment was focused on paraphyses, septate orientation, spore, asci and number of ascospores, and aspic. Images were taken with an Olympus microscope (Olympus Ltd., Nanjing China) at 40× and 100× magnifications.

### DNA extraction

To obtain pure mycelium, ascospores ejected from the fruit bodies were cultured on Potato Dextrose Agar (PDA) medium (200 g potato, 20 g dextrose, and 20 g agar per 1 L deionized water) until a putative colony developed. The colony was isolated and purified on a new petri dish with PDA medium and was then used for future molecular phylogenetic analysis.

Mycelia grown for two weeks on PDA dishes were collected into a 1.5 mL tube and then ground with quartz sand using a hand grinder. DNA extraction was performed using the CTAB method described by^12,15^

### PCR amplification and sequencing

All extracted DNA samples were used as substrates of PCR amplification with five pairs of partial gene datasets. PCRs were performed in a total volume of 20 µL containing 1–2 µL template DNA, 10 µL of 2 × Ex Taq Master mix (Ex Taq DNA polymerase, 3 mM MgCl_2_, and 400 µM of each dNTP), 1 µL of each primer, and sterilized distilled water until a total of 20 µL was reached. PCR products were obtained using a Bioer Cycler machine (Bioer Technology Co. Ltd., Hangzhou, China). The cycling parameters of the PCRs are shown in Table 3. Amplicons were analysed in 1% agarose gel electrophoresis by using 0.05 × TBE buffer complemented with 2 µL ethidium bromide. The size of the DNA band was visualized with a UV transilluminator. PCR products were purified and sequenced by Aoke Biotech Co., Ltd. (Yangling, China). All raw sequences were assembled and edited using the Bioedit software version 7.0 9.0^33,34^ Clean sequences were deposited in GenBank (NCBI) under the accession numbers shown in Table 2.

**Table 3:** Primer pairs used in this study.

Primers	Sequences	Annellation	References
ITS1 F	5′-TCC GTA GGT GAA CCT GCG G-3′	58–60 °C	^18,39^
ITS4 R	5′-TCC TCC GCT TAT TGA TAT GC -3′		
LROR F	5′- ACC CGC TGA ACT TAA GC-3′	56–57 °C	^21^
LR5 R	5′- ATC CTG AGG GAA ACT TC **-**3′		
EF1–526 F	5′-GTC GTY ATY GGH CAY GT-3′	58–59 °C	^40^
EF1-3A R	5′- GAA ACG RTC CTC RGA CCA C-3′		
PBB1-A F	5′-GTC CGG GWC ATT TTG GTC-3′	59–60 °C	^23^
RPB1-C R	5′-TTG TCC ATC TAN GTR GCR ACA-3′		
RPB2-6 F	5′-TGG GGY ATG GTN CCY GC-3′	60–61 °C	^24^
RPB2-7.1 R	5′-CCC ATR GCY TGY TTM CCC ATD GC-3′		^25^

### Phylogenetic analysis

Raw sequences of the 38 collections were individually revised, and their ends were trimmed using the Bioedit software version 9.0^33,34^. Multiple sequence alignment of single genes were performed using ClustalW implemented in the MEGA 7 software under the full processing mode^35^, to establish the position of the nucleotides. Multiple sequence alignment of the concatenated gene sequences was performed using MAFFT implemented in the UGENE software (Unipro, Russian). The aligned sequences, including those of previous studies obtained from GenBank and MLST^10–12,26^, were manually adjusted when necessary, gaps and ambiguously aligned nucleotide positions in *EF*, *RBP* sequences were excluded from the datasets. Phylogenetic trees of single genes and multigene combinations were constructed using the maximum-likelihood method in MEGA 7.0 under the GTR + I model of evolution with 1,000 bootstrap replicates^36–38^

## Supplementary information

Supplementary information
